This article has been retracted.

# A Real-Time Crowd Monitoring and Management System for Social Distance Classification and Healthcare Using Deep Learning

**DOI:** 10.1155/2022/2130172

**Published:** 2022-04-05

**Authors:** Sangeeta Yadav, Preeti Gulia, Nasib Singh Gill, Jyotir Moy Chatterjee

**Affiliations:** ^1^Department of Computer Science & Applications, Maharshi Dayanand University, Rohtak, India; ^2^Department of Information Technology, Lord Buddha Education Foundation, Kathmandu, Nepal

## Abstract

Coronavirus born COVID-19 disease has spread its roots in the whole world. It is primarily spread by physical contact. As a preventive measure, proper crowd monitoring and management systems are required to be installed in public places to limit sudden outbreaks and impart improved healthcare. The number of new infections can be significantly reduced by adopting social distancing measures earlier. Motivated by this notion, a real-time crowd monitoring and management system for social distance classification is proposed in this research paper. In the proposed system, people are segregated from the background using the YOLO v4 object detection technique, and then the detected people are tracked by bounding boxes using the Deepsort technique. This system significantly helps in COVID-19 prevention by social distance detection and classification in public places using surveillance images and videos captured by the cameras installed in these places. The performance of this system has been assessed using mean average precision (mAP) and frames per second (FPS) metrics. It has also been evaluated by deploying it on Jetson Nano, a low-cost embedded system. The observed results show its suitability for real-time deployment in public places for COVID-19 prevention by social distance monitoring and classification.

## 1. Introduction

Coronavirus has shaken the whole world after being first observed in China. Its symptoms comprise shortness of breath, fever, chills, loss of taste and smell, body aches, and cough. Coronavirus is primarily spread by physical contact. Its first case was discovered in Wuhan, China, in December 2019. After some time, it spread its roots in the whole world and resulted in a pandemic that has caused a number of infections comprising many fatalities. To save the life of the masses, severe lockdowns were imposed in various countries. The vaccination efforts and preventive measures have contributed a lot to control its spread. The industries, workplaces, and travel are returning to their normal state. But due to the mutations in this virus, a number of new variants are emerging. The WHO (World Health Organization) has also declared this disease as pandemic due to its fatality and severity. The complexities and eruption of new variants have made the spread and duration of this virus unpredictable. No vaccine with full efficacy has been developed yet [1]. It can only be prevented by maintaining social distancing, frequently washing hands, and wearing masks. As it spreads fast by close contact, the infected people are quarantined either in their homes or in hospitals to prevent its further spread to others. To mitigate its mass spread, the nations had to impose lockdown, close their boundaries, stop public gatherings, and close schools, colleges, and workplaces. It has been observed that the adoption of such strict measures has resulted in a reduced number of infections and fatalities [2].

It has also been reported that fever is the primary symptom of this virus, and studies in China also found that 99 percent of the infected people are found to have a high temperature. To measure a person's surface temperature, noncontact infrared thermometers and thermal cameras are being used. This massive move significantly limits the widespread of this virus.

According to WHO, social distancing is the most significant preventive measure where people can keep a certain distance from one another, hence minimizing physical contact from virus carriers. The employment of technological tools for the enforcement of social distancing is of main concern. ICT (Information and Communications Technology) and Artificial Intelligence tools could play a significant role in addressing this challenge of implementing social distancing practice. The application of Artificial Intelligence tools can help in prior identification of the infections and diagnosing the same with AI-equipped tools and medical imaging techniques. To predict and monitor the spread of this disease automatically, a number of intelligent neural network-based networks have been designed. Moreover, AI is also helpful in contact tracing by identifying hotspots and clusters. AI tools can also be utilized in finding the most sensitive places and people so that preventive measures can be taken accordingly. In this way, AI is playing an important role in imparting more preventive and predictive healthcare.

Social distancing is the primary prevention measure to lessen the mass spread of this virus. Motivated by this notion, a real-time crowd monitoring and management system is proposed to detect the social distancing in the common places, hence imparting improved healthcare by reducing the number of infections. The system utilized the YOLO v4 person detection and Deepsort technique along with a social distancing classification algorithm.

The paper is organized as follows. Research background and related work have been detailed in Section 2. The details of the proposed system have been given in Section 3.  Section 4 contains the experimental results and their analysis. The whole work is concluded in Section 5.

## 2. Research Background

The temperature screening and social distancing are effective preventive measures in mitigating the mass spread of the coronavirus. These are highly recommended by World Health Organization and several other medical organizations [3]. The efficacy of social distancing on the transmission of this virus has been studied by Russel et al. [4]. They have presented the trajectory of the outbreak produced by scientific location contact patterns employing SEIR, that is, susceptible exposed infected removed techniques. It has also been presented that sudden removal of social distancing could result in a wider spread of the infection. The effect of social distancing on other genres has been studied and presented by Nabil Kahale [5]. The main motive of this research is to present an approximation showcasing how new infections and economic loss can be significantly reduced by early social distancing. During the coronavirus outbreak, the researches majorly focused on finding and developing efficient measures to diminish its spread among society [6, 7]. Technological advancements could play a prominent role in preventing its mass spread by detecting infected people at the earliest. A COVID-19 infected person can be tracked via GPS and smartphones' enable applications [8]. This technology has limited applicability and cannot be used to track people who do not have cell signals or Wi-Fi. Moreover, the mass gatherings in the open space can be tracked using drones employed with video cameras [9, 10]. Such technological advancements could help curb or prevent the outbreak.

The advancements in the computer vision domain and deep learning have made the task of classification and object detection solvable and easier. These researches contributed to different genres of vision comprising segmentation, neural style transfer, and object tracking in addition to detection [11].

Deep Learning, an important branch of Artificial Intelligence, evolved as a significant tool for object detection and data processing. Primarily deep learning comprises sophisticated neural network design. Its concept originated back ago in the 1940s [12]. The learning problems can be solved efficiently with such neural network designs [13]. CNN- (Convolutional Neural Network-) based object detection models are widely used. These networks take an image as an input, and the learnable biases and weights are given to the different classes in the image and accordingly distinguish them from each other. The advancements in CNN networks made their augmentation possible with low complex low-resolution input-based embedded systems. A number of object detection techniques based on different deep learning models like YOLO, Single-Shot Detector (SSD), and R-CNN are available these days. These algorithms are based on efficient motion estimation in the video stream. An efficient technique of person detection in the video stream has been proposed by Ebrahim et al. [14]. The technique comprises a deep learning person detector employed with Gaussian mixture and background subtraction. Another method of person detection has also been presented in [15]. Here, an amalgamation of machine learning and deep learning methods is utilized to attain more precise results with less computation. But this model slows down when used in real-time detection-based applications. The researchers have also proposed a model to detect static crowds [16]. In this method, the mean is taken as SVM (Support Vector Machine) for the categorization of the spots as the groupings of the people. The text features then extract these grouping spots. A pedestrian detection system is proposed in [17], which detects the walking person by background subtraction and then makes the real-time classification. Similar works pertaining to smart cities have also been carried out in [18, 19]. To track the objects in a scenario, a number of deep learning-based tracking techniques like POI (Person Of Interest), SORT (Simple Online and Real-Time Tracking), and EMATT (Expendable Mobile ASW Training Target) have also been proposed. These techniques present variation in their results based on the different performance metrics taken.

Keeping in view the limitation of different techniques, a novel real-time crowd monitoring and management system is proposed for imparting improved healthcare by monitoring the social distance among people in the common places utilizing YOLO v4 and Deepsort techniques for person detection and their tracking.

## 3. Overview of Object Detection

The object detectors detect an object by putting a bounding box and then assign its corresponding label. Deep learning-based object detection has outperformed all earlier traditional schemes and is now widely used for object detection and classification tasks. An efficient deep learning-based detector, R-CNN, that is, Regional Convolutional Neural Network, is proposed by Girshick [20]. This network works in four steps. Firstly, the picture is given as an input to the detector, and then regional proposals are extracted. The CNN computes the features of the extracted region proposals and classifies them. The schematic diagram of the same has been given in Figure 1, depicting the whole process of detection and classification by R-CNN.

The region proposals are extracted using selective search algorithms. This process is time-consuming, approx. taking 47 seconds to perform regional classifications of each image, hence not suitable for real-time applications. Moreover, this network cannot be end-to-end trained, but each part has to be trained separately.

To overcome the disadvantage of the above R-CNN, the same author has proposed its fast variant, Fast R-CNN [21]. Its basic working algorithm is the same as of R-CNN, but some changes are made to make faster detection. In this model, the input image is given to a CNN, which then generates a convolutional feature map of the same. ROI (Region of Interest) pooling layer is utilized to reshape the squared regions into a fixed size. These regions are then fed to the softmax employed FC (Fully Connected) layer for predicting the label of the region.  Figure 2 presents the design of the R-CNN detector.

To extract the region proposals, selective search algorithms are used by Fast R-CNN. These algorithms are time-consuming and slow, hence affecting the overall performance of the detection network.

YOLO emerged as one of the efficient object detectors based on deep learning. Recent advancements result in its various versions, including YOLO v2, v3, and v4. YOLO was initially proposed by Redmon et al. [23]. For a whole image, this technique utilized a single neural network. The input image to this network is segregated into different partitions. Each region is then surrounded by a bounding box, and corresponding probabilities are computed. YOLO scans the full image in a single time, and hence, the predictions are informed by the image context. Unlike R-CNN, YOLO works with a single network evaluation. It divides the input image into SxS grids, and then the features are extracted individually from them. The bounding boxes are predicted along with their corresponding labels. These labels are associated with their predicted confidence score. This process of object detection and prediction is depicted in Figure 3.

YOLO predicts the confidence score of all bounding boxes detected from the grid cells. The predictions of the bounding box are represented by five parameters, namely, *w*, *h*, *x*, and *y*, along with the confidence score. The height of the image is given by *h* and *w* presents the width of the same. The center of the bounding box is represented by (*x,y*) parameters. The confidence score provides the confidence of the detector for the predicted object.

A number of bounding boxes are predicted for every grid cell. In YOLO, during the training phase, only one predictor per bounding box is required. For the ground truth estimation, the detector is trained to predict the object with the highest IoU (Intersection over Union) value. It leads to the more specialized bounding box prediction. The sum squared error between the predicted and actual classes is used for the loss estimation, and henceforth localization, classification, and confidence loss are computed for the network. Equation (1) presents the loss function used by YOLO to enhance and optimize its performance during the training phase.

(1) $$\begin{array}{c} \lambda_{\text{coord}}\sum_{i=0}^{s^{2}}1_{i,j}^{\text{obj}}\left[{\left(x_{i}-{\hat{x}}_{j}\right)}^{2}\right]\\ +\lambda_{\text{coord}}\sum_{i=0}^{s^{2}}\sum_{j=0}^{B}1_{i,j}^{\text{obj}}\left[{\left(\sqrt{w_{i}}-\sqrt{{\hat{w}}_{i}}\right)}^{2}+{\left(\sqrt{h_{i}}-\sqrt{{\hat{h}}_{i}}\right)}^{2}\right]\\ +\sum_{i=0}^{s^{2}}\sum_{j=0}^{B}1_{i,j}^{\text{obj}}{\left(\sqrt{C_{i}}-\sqrt{{\hat{C}}_{i}}\right)}^{2}+\lambda_{\text{coord}}\sum_{i=0}^{s^{2}}\sum_{j=0}^{B}1_{i,j}^{\text{noobj}}{\left(\sqrt{C_{i}}-\sqrt{{\hat{C}}_{i}}\right)}^{2}\\ +\sum_{i=0}^{s^{3}}1_{i}^{\text{obj}}\sum_{c\in \text{ class}}\left(p_{i}\left(c\right)-{\hat{p}}_{i}{\left(c\right)}^{2}\right), \end{array}$$

where the following parameters are used as follows: ℷ _coord_ is a constant value used to increase the weight for the first two terms of the loss function, ℷ _noobj_ is used to weigh down the loss when detecting the background, *S*^*2*^ is the number of cells, *B* is the number of box predictions for each cell, 1_*i*,*j*_^obj^ is one if there is an object in cell *i* and among all the predictors of this cell, the confidence of *j*^*th*^ predictor is the highest, *x*_*i*_ and *y*_*i*_ are the anchor box's centroid, *w*_*i*_ is the anchor box's width, *h*_*i*_ is the anchor box's height, *C*_*i*_ is the confidence score, ∧*Ci* is the box *j*'s confidence score in cell *i*, 1_*i*,*j*_^noobj^1_*i*,*j*_^obj^ complement of *1*_*i*_^*obj*^ is one if an object is found in cell *i*, otherwise zero, *p*_*i*_*(c)* is the classification loss, and ∧ *p*_*i*_*(c)* is the class *c*'s conditional class probability in cell *i*.

YOLO v2, v3, and v4 are the subsequent versions of YOLO. Several enhancements and improvements are made for real-time processing [24, 25]. The later versions resulted in a faster network along with significant accuracy improvement. Batch normalization is employed in all CNN layers to address the localization errors. YOLO v4 is the most recent version of YOLO [26]. It comprises three components, namely, the backbone network component, neck component, and prediction head component. The backbone component plays an important role in input dimension reduction and translation to more complex features. The schematic diagram of the same is given in Figure 4.

We have used the CSPDarknet53 backbone for our implementation. The neck component takes features from the backbone network and mixes them. It can consist of components like Spatial Pyramid Pooling (SPP) and Path Aggregation Network (PANet). It results in better spatial information preservation and extracting features at various resolutions. For the single-stage prediction head of YOLO, the bounding boxes to the detected objects are created using anchor boxes. These anchor boxes have predefined width and height and are rectangular in shape. The size of bounding boxes of the objects present in the training dataset determines the height and width of anchor boxes.

## 4. Proposed System

Deep learning's emergence has offered the finest performing algorithms for the different problems and tasks pertaining to diverse domains, including object detection and tracking, medical diagnosis, and much more. A crowd monitoring and management system is proposed to impart improved healthcare using deep learning techniques to monitor and detect social distancing in public places. To maintain a balance of precision and speed, YOLO v4 and Deepsort techniques are used. People are predicted using bounding boxes around each detected object. The circle of influence is calculated for each person. Later, all circles of influence are accumulated for a frame and those having more overlap locations result in high intensity. The result of each surveillance frame is color-coded, depicting the statistical density of people. The details of the whole system regarding social distance detection, network design, Deepsort-based tracking, and algorithm for distance classification are given in the following subsections.

### 4.1. Detection of Social Distance

The process of detection of social distance from the video stream captured using the cameras installed in public places comprises the following steps, and the corresponding flowchart is given in Figure 5:

1. The video stream is prepared from a camera, and it comprises people.
2. People in images or video streams are detected using a deep learning object detector.
3. Track the detected people using a Deepstream-based tracker.
4. Calculate the circle of influence for each detection.
5. Compute the overlap between the circle of influence of the detected people to identify a breach of social distancing.
6. Aggregation of overlap results in a heatmap-like image with a higher crowd resulting in higher intensity. It can be used to identify violations and hotspots and generate real-time alerts.

Algorithm for social distance detection. The following algorithm is used for the detection of social distance and finally generating alerts accordingly seeing the intensity of breach:

1. Input image stream is taken from the installed camera.
2. People are extracted from images using a YOLO v4 object detector.
3. Detected people are tracked using the Deepstream-based tracker.
4. Circle of influence of each detection is calculated.
5. Overlap among the circle of influences has been determined.
6. Intensity of breach of social distance has been identified.
7. Real-time alerts are generated.

### 4.2. Neural Network Design

The original YOLO v4 comprises SPP module, CSPDarknet53 backbone, and anchor-based detection head along with PANet path-aggregation neck. A 725 × 725 receptive field, 29 convolutional layers of size 3 × 3, and 27.6 M parameters are used in CSPDarknet53. The computation of such a network is quite expensive. Hence, we have used a lightweight model variant YOLO v4-tiny to achieve desired goals. The input layer of the system fed the images of size (416 × 416 × 3) to the network. It contains an optimized CSP backbone with fewer layers and parameters. The Spatial Pyramid Pooling (SPP) or equivalent, Fast Spatial Pyramid Pooling (SPPF) block, is utilized over the CSPDarknet53 to extract the most notable context features, to enhance the receptive field without any compromise with the speed. The parameter aggregation from the diverse backbone and detection levels is achieved using the PANet method. Finally, pyramid features are processed by the detection head to provide the detection.  Figure 6 depicts the design of the YOLO v4-tiny neural network.

### 4.3. Deepsort-Based Tracking

Deepsort is an efficient deep learning-based technique used for tracking objects in videos. The proposed system utilizes Deepsort to track the detected people in the video stream. To predict trajectories of the objects, the learned patterns from the identified objects in the images are coupled with the temporal information. Each object is tracked by assigning a unique ID, and these IDs mapped to the objects of interest are utilized for future statistical analysis. The several issues pertaining to object tracking like nonstationary cameras, numerous views, occlusion, and annotating training data are effectively addressed by the Deepsort. The Hungarian algorithm and the Kalman filter are used for accurate tracking. For the enhanced association and prediction of future locations of the object, the Kalman filter is recursively used. Along with association, the Hungarian method is employed for ID attribution and for identifying the same object in the current and past frame. A linear constant velocity Kalman filter model is used for tracking, and the corresponding target object to be tracked is described with eight dimensions, as presented by equation (2).

(2) $$\begin{array}{c} x=\left[x^{\prime },y^{\prime },u,v,\lambda^{\prime },h^{\prime },\lambda ,h\right], \end{array}$$

where *x* is the target object, *(u, v)* is the centroid of the bounding box, *h* is the video height, and *λ* is the aspect ratio.

The variables' respective velocities are represented by the other variables. Later, a Kalman filter is utilized where *u, v, λ,* and *h* parameters are used as the bounding coordinates for the object state. The total number of frames is determined for each track *k*, beginning with the most recent successful measurement connection. When the Kalman filter predicts a positive result, the counter is increased, and when the track is connected with a measurement, the counter is reset to 0. If the recognised tracks are older than a predetermined limit, those items are judged to leave the scenario, and the corresponding track is removed from the collection.  Table 1 compares the accuracy and speed of Deepsort in object tracking. The comparison uses metrics like multiobject tracking precision (MOTP), multiobject tracking accuracy (MOTA), mostly tracked (MT) as tracks with more than 80% tracking, mostly lost (ML) as tracks with less than 20% tracking, identity switches (ID), and fragmentation (FM). ID is the number of times ground truth identity changes. FM gives a count of interruptions due to missing detection.

### 4.4. Algorithm for Distancing Classification

The proposed system classifies and decides the safe distancing among the detected people and then represents this information in a visual manner. The top view of the scene is required to compute the distance between the people. In the standard approach for distance classification, the distance between people is measured by the distance between each detected person bounding box. The proposed system employs a novel approach for monitoring social distancing in a crowded scene. In this approach, the unsafe social distancing is represented by the red color bounding box, and the rest of the colors denote the safe distancing. A screenshot of the same has been given in Figure 7. Firstly, the total number of people in an image is identified. If the number of people's bounding boxes exceeds two, the distance between them is calculated by the gap among the centers of their corresponding bounding boxes. Equation (3) presents *CP(x,y),* center point computation of the bounding box.

(3) $$\begin{array}{c} \text{CP}\left(x,y\right)=\left(\left(X\min+X\max\right)/2,\left(Y\min+Y\max\right)/2\right), \end{array}$$

where the given parameters denote the different dimensions of the bounding box as follows: *CP* is the center point, *Xmin* is the bounding box's width, minimum value, *Ymin* is the bounding box's height, minimum value, *Xmax* is the bounding box's width, maximum value, and *Ymax* is the bounding box's height, minimum value.

The Euclidean formula is used to compute the distance among the centers of bounding boxes. Here, the distance between pixels is transformed into a metric distance which is then compared to the threshold value. If this computed value is less than the threshold value, such boxes will appear in red color. Otherwise, they will appear in different colors. The distance among people can be effectively computed with the top view of the scene, and this is achieved by homographic transformation of the concerned scene. To map with the real-world distance between people, this computed space is scaled by a scaling factor S, and it is determined by the number of pixels of the image corresponding to one meter in the real world.

The system focuses on identifying bad actors who are breaching the social distance and taking action on them. Real-time monitoring and acting on people on a large scale poses different types of social, operational, privacy, and morale-related challenges. Also, given the size and changing nature of bounding boxes in a video frame, it is difficult to monitor this in real time. To address the above concerns, we implemented a novel social distance monitoring method that focused more on the system or physical structure where the breach was happening and incentivised to improve the system. We represent the physical system in a color-coded heatmap where the breach is happening and what is the severity of the breach. The corresponding screenshots have been given in Figures 8 and 9.

To obtain the structural heatmap of the social distancing breach, first, the circle of influence for each tracked bounding box is calculated. It is calculated by scaling the corresponding bounding box with a scaling factor S, which is determined by the number of pixels of the image corresponding to one meter in the real world. Then, the overlap between the circles of influence of the detected people is computed to identify a breach of social distancing. Finally, overlap frames are aggregated over a time window of T seconds. Aggregation of overlap results in a heatmap-like image with a higher crowd resulting in higher intensity. It can be used to identify violations and hotspots and generate real-time alerts.

## 5. Experimental Results

We have used two different datasets for evaluating the performance of the system. For testing the accuracy and performance of different object detection techniques for person detection tasks, a standard MS-COCO dataset is used. It comprises 1.5 million annotations of 80+ object categories. It is one of the standard datasets used for benchmarking object detection. In order to test the end-to-end application with tracking and social distance heatmap visualisation, we have used the surveillance footage of the Oxford town center. This video contains 7500 frames annotated with person category.

Figure 10 presents the comparative results of the performance of YOLO v4 with other object detectors. For the MS-COCO dataset, it reports 43.5% AP with ∼65 FPS on Tesla V100.

The experimental results of models evaluated with mAP are given in Table 2. For faster R-CNN evaluation, we resized images to a resolution of 600 × 600 pixels by scaling shorter dimensions to 600 pixels and then taking a center-crop of size 600 × 600 pixels. The images are scaled to 416 × 416 pixels with fixed dimensions in YOLO. The maximum mAP with the lowest FPS has been observed with a faster R-CNN model. The required model should have high enough accuracy with low compute requirements to make it suitable for real-time operation on embedded devices. Low-performance results make the faster R-CNN model not suitable for real-time applications. The performance of YOLO v3 and YOLO v4-tiny is the highest, meeting the real-time application requirements. Compared to YOLO v3-tiny, YOLO v4-tiny shows better results with balanced FPS and mAP score and hence used for social distance detection among people in the surveillance video.

YOLO v4-tiny is approximately 8 times as fast at inference time as YOLO v4 as per the performance metrics, and on a very hard MS-COCO dataset, its performance is about two-thirds. If only person detection tasks are concerned, where people are readily visible in CCTV camera, there is even less performance degradation.

### 5.1. Jetson Based Real-Time Implementation Statistics

For large-scale implementation, the algorithm needs to be deployed on low-cost embedded devices such as Jetson Nano, TX2. We selected only YOLO variants for the implementation because of their higher performance combined with good accuracy. For benchmarking, we selected Jetson Nano and Jetson TX2 platforms. The FPS for YOLO v3 and YOLO v4 models in full and tiny variants on different scales of images during real-time detection with embedded SOCs have been given in Table 3.

After careful evaluation, YOLO v4-tiny is selected in our final implementation for person detection at 416 × 416 resolutions and then combined with Deepsort for tracking and our social distance monitoring approach. Our system achieved end-to-end performance of 6 FPS on Jetson Nano which met the requirement of real-time monitoring of social distancing. Jetson Nano is also very power efficient, consuming only 5.4 W while displaying distancing heatmap on a monitor.  Table 4 depicts the power usage of Jetson Nano at different configurations.

For achieving improved healthcare by adopting social distancing measures earlier, the large-scale infrastructure for social distance monitoring is required, comprising edge cameras and computing units to be installed at the public spaces with a communication network for central monitoring. This kind of large-scale public space automatic monitoring can play an essential role in mitigating the spread and impact of subsequent COVID-19 waves. Since this application is intended to be used in public spaces with various environmental and lighting conditions, high end-to-end accuracy is required. Along with the accuracy of the system, the privacy and individual rights of observed people are also a genuine concern. The system should not disclose a person's identity in general and should not assist in targeted tracking and surveillance of common people. Maintaining transparency about its fair uses by its stakeholders is also very essential.

## 6. Conclusion

The paper proposes a real-time crowd monitoring and management system for imparting improved healthcare by social distance detection and classification in public places using deep learning-based YOLO v4 object detection and Deepsort techniques. The bounding box generated around people helps in detecting the groups, and their closeness is computed with the help of the circle of influence approach. The system also generates a color-coded heatmap of physical structure depicting where the breach of social distancing is happening and what is the severity of the breach. The proposed system has also been deployed, tested, and evaluated on Jetson Nano, a low-cost embedded system to meet the requirements of real-time large-scale deployments. The observed results show the suitability of this system in COVID-19 prevention in public places by social distance detection and classification via crowd monitoring in real time [27–30].

## Figures and Tables

**Figure 1:** The working of the R-CNN detector.

**Figure 2:** Network design of Fast R-CNN [22].

**Figure 3:** Object detection by YOLO.

**Figure 4:** YOLO v4 object detection architecture.

**Figure 5:** Steps followed to measure social distancing.

**Figure 6:** YOLO v4-tiny neural network.

**Figure 7:** Screenshot of person detection by the proposed system.

**Figure 8:** Screenshot of social distance measured by the proposed system.

**Figure 9:** Red area shows the breach of social distance as measured by the proposed system.

**Figure 10:** Performance analysis of YOLO v4 over the MS-COCO dataset.

**Table 1:** Comparative results of Deepsort with other techniques.

	Deepsort (ours)	POI	SORT	EAMTT
MOTA	61.4	66.1	59.8	52.5
MOTP	79.1	79.5	79.6	78.8
MT	32.8%	34.0%	25.4%	19.0%
ML	18.2%	20.8%	22.7%	34.9%
ID	781	805	1423	910
FM	2008	3093	1835	1321
FP	12852	5061	8698	4407
FN	56668	55914	63245	81223
Runtime	40 Hz	10 Hz	60 Hz	12 Hz

**Table 2:** Performance comparison of various object detectors.

Detection models	Object detection accuracy (AP50)	F (%) PS (1080Ti)
Faster R-CNN	73.2	6
MobileNet SSD V2	33.7	380
YOLO v3	58.5	90
YOLO v3-tiny	34.8	360
YOLO v4	64.9	75
YOLO v4-tiny (proposed)	40.2	300

**Table 3:** FPS for YOLO v3 and YOLO v4 model in full and tiny variants on different scales of images during real-time detection with embedded SOCs.

DL model	Nvidia Jetson Nano		Nvidia Jetson TX2	
Input size ->	**416**	**608**	**416**	**608**
YOLO v3	3	1.5	6.4	3
YOLO v4	2.5	1.3	6.7	3.8
YOLO v3-tiny	15	5.2	20	12
YOLO v4-tiny^*∗*^	10	7	15	9.5

**Table 4:** Measurement of power consumption.

	Jetson Nano without monitor, keyboard, and mouse		Jetson Nano with monitor, keyboard, and mouse	
Algorithm status	Off	Running	Off	Running
Power measurement (W)	1.24	4.40	2.24	5.40

## Data Availability

The data are available upon request from the authors.
